The article "Identification of 5 Hub Genes Related to the Early Diagnosis, Tumour Stage, and Poor Outcomes of Hepatitis B Virus-Related Hepatocellular Carcinoma by Bioinformatics Analysis" was published in 2021. Journal: Comput Math Methods Med.

# Identification of 5 Hub Genes Related to the Early Diagnosis, Tumour Stage, and Poor Outcomes of Hepatitis B Virus-Related Hepatocellular Carcinoma by Bioinformatics Analysis

**DOI:** 10.1155/2021/9991255

**Published:** 2021-09-23

**Authors:** Rui Qiang, Zitong Zhao, Lu Tang, Qian Wang, Yanhong Wang, Qian Huang

**Affiliations:** ^1^Department of Infectious Diseases, Guang'anmen Hospital, China Academy of Traditional Chinese Medicine, Beijing 100053, China; ^2^Department of Oncology, The Second Affiliated Hospital of Harbin Medical University, Harbin 150081, China; ^3^Department of Traditional Chinese Medicine, Kunming Second People's Hospital, Kunming, 650000 Yunnan, China; ^4^Department of Basic Medicine, Yunnan University of Business Management, Kunming, 650000 Yunnan, China; ^5^Department of Second Internal Medicine, Chongming Branch of Yueyang Integrated Hospital of Traditional Chinese and Western Medicine Affiliated to Shanghai University of Traditional Chinese Medicine, Chongming, 202150 Shanghai, China; ^6^Department of Oncology, Shanghai Xinhua Hospital Chongming Branch Affiliated to Shanghai Jiaotong University School of Medicine, 25 Nanmen Road, Chengqiao Town, Chongming District, 200000 Shanghai, China

## Abstract

**Background:**

The majority of primary liver cancers in adults worldwide are hepatocellular carcinomas (HCCs, or hepatomas). Thus, a deep understanding of the underlying mechanisms for the pathogenesis and carcinogenesis of HCC at the molecular level could facilitate the development of novel early diagnostic and therapeutic treatments to improve the approaches and prognosis for HCC patients. Our study elucidates the underlying molecular mechanisms of HBV-HCC development and progression and identifies important genes related to the early diagnosis, tumour stage, and poor outcomes of HCC.

**Methods:**

GSE55092 and GSE121248 gene expression profiling data were downloaded from the Gene Expression Omnibus (GEO) database. There were 119 HCC samples and 128 nontumour tissue samples. GEO2R was used to screen for differentially expressed genes (DEGs). Volcano plots and Venn diagrams were drawn by using the ggplot2 package in R. A heat map was generated by using Heatmapper. By using the clusterProfiler R package, KEGG and GO enrichment analyses of DEGs were conducted. Through PPI network construction using the STRING database, key hub genes were identified by cytoHubba. Finally, KM survival curves and ROC curves were generated to validate hub gene expression.

**Results:**

By GO enrichment analysis, 694 DEGs were enriched in the following GO terms: organic acid catabolic process, carboxylic acid catabolic process, carboxylic acid biosynthetic process, collagen-containing extracellular matrix, blood microparticle, condensed chromosome kinetochore, arachidonic acid epoxygenase activity, arachidonic acid monooxygenase activity, and monooxygenase activity. In the KEGG pathway enrichment analysis, DEGs were enriched in arachidonic acid epoxygenase activity, arachidonic acid monooxygenase activity, and monooxygenase activity. By PPI network construction and analysis of hub genes, we selected the top 10 genes, including CDK1, CCNB2, CDC20, BUB1, BUB1B, CCNB1, NDC80, CENPF, MAD2L1, and NUF2. By using TCGA and THPA databases, we found five genes, CDK1, CDC20, CCNB1, CENPF, and MAD2L1, that were related to the early diagnosis, tumour stage, and poor outcomes of HBV-HCC.

**Conclusions:**

Five abnormally expressed hub genes of HBV-HCC are informative for early diagnosis, tumour stage determination, and poor outcome prediction.

## 1. Introduction

Most primary liver cancers among adults worldwide are hepatocellular carcinomas (HCCs, or hepatoma) [1], and HCCs are the 3rd leading cause of cancer-associated deaths [2]. HCC generally develops from chronic liver diseases such as chronic hepatitis B/C virus (HBV or HCV) infection, alcohol abuse liver disease, nonalcoholic fatty liver disease (NAFLD), and cirrhosis [3]. Chronic hepatitis infection is the main cause of the pathogenesis of HCC in sub-Saharan Africa (SSA) and East Asia [4, 5]. Chronic hepatitis infection with HBV is a well-known risk factor for HCC metastasis or recurrence [6]. For early-stage HCC patients, curative surgery is the predominant treatment option [7]. For inoperable tumours and tumour relapses after surgery, the preferred alternatives are chemotherapy, radiation therapy, and targeted therapy [8]. Unfortunately, not all patients benefit from conventional medical therapy. Although aggressive therapy measures are used, patients with advanced HCC have a poor prognosis [9]. Thus, an improved understanding of the underlying mechanisms of pathogenesis and carcinogenesis at the molecular level for this cancer could facilitate the development of novel early diagnostic and therapeutic treatments to improve the approaches and prognosis of HCC patients.

During the last several years, with rapid advances in bioinformatics tools and high-throughput sequencing technologies [10], such as microarrays and next-generation sequencing (NGS), a general view of the occurrence, development, and metastasis of various types of cancers is possible. Specifically, widely used high-throughput platforms can be applied to prediction screening, early diagnosis, prognosis, and individualized prevention and therapy [11–15]. Differentially expressed genes (DEGs) and noncoding RNAs (ncRNAs), which include microRNAs, small interfering RNAs (siRNAs), long noncoding RNAs, circular RNAs, and differentially methylated CpG sites, may provide valuable information for the survival prediction of HBV-associated HCC (HBV-HCC). However, a number of factors, such as sample heterogeneity, diverse screening methods, diverse data mining techniques, and the coupling effect of limited sample size in a single independent study, may generate false-positive and false-negative findings. To overcome these limitations, integrated analysis based on collective datasets has been identified as a promising alternative. Hence, many recent studies have successfully used public datasets, such as The Cancer Genome Atlas (TCGA), Gene Expression Omnibus (GEO), and International Cancer Genome Consortium (ICGC), to identify new diagnostic and prognostic molecular markers to treat cancer [16–20]. Thus, database mining and analysis have become essential first steps for a wide range of applications in molecular biology. At present, reports about HBV-HCC dysregulated genes and HBV-HCC candidate biomarkers that can be combined with microarray datasets in the literature are scarce. Therefore, to provide a new basis for diagnosis and treatment, a comprehensive, whole-genome analysis of microarray datasets must be adopted.

For this purpose, we first explored the key DEGs associated with HBV-HCC by bioinformatics analysis of the GEO database and TCGA. This was followed by Gene Ontology (GO) functional and Kyoto Encyclopedia of Genes and Genomes (KEGG) pathway enrichment analysis of DEGs,

The predicted protein–protein interaction (PPI) network was constructed by using the Search Tool for the Retrieval of Interacting Genes (STRING; https://string-db.org/) database. Within this, the hub genes were screened. Next, we evaluated the clinical cancer staging value and prognostic value of the hub genes in TCGA. Finally, key hub genes were identified and validated using immunohistochemistry in the Human Protein Atlas database (THPA, https://www.proteinatlas.org/). Taken together, this paper had two main purposes. The first purpose was to elucidate the molecular mechanism by which HBV contributes to HCC development and progression. The second purpose was to screen the indicated genes to identify reliable early diagnostic and prognostic biomarkers and therapeutic markers.

## 2. Methods

### 2.1. Microarray Data

We downloaded GSE55092 and GSE121248 gene expression profiling data, which had not been previously studied simultaneously, from the Gene Expression Omnibus (GEO) database (https://www.ncbi.nlm.nih.gov/geo/).

The chip-based platform GPL570 (HG-U133_Plus_2) Affymetrix Human Genome U133 Plus 2.0 Array was applied for the mRNA expression profiling of both databases. The GSE55092 dataset, containing 49 HCC samples and 91 nontumour tissue samples, was obtained at various distances from the tumour centre in individual livers of 11 HBV-associated HCC patients [21]. The GSE121248 dataset, containing 70 HCC samples and 37 nontumour tissue samples, was obtained from chronic hepatitis B-induced HCC and their adjacent normal tissues [22]. This study was not conducted on human biological specimens, and two sets of microarray data were downloaded from the GEO database. Thus, according to Chinese law, this research did not require an ethical review board or committee approval or patient consent.

### 2.2. Identification of DEGs

GEO2R (https://www.ncbi.nlm.nih.gov/geo/geo2r) is an R-based interactive web tool and was used to screen for DEGs between HCC and nontumour tissues. Based on the significance threshold of adj.*P* value < 0.05 and logFC > 1 (upregulated) or logFC < −1 (downregulated), the significantly DEGs were identified. Volcano plots and a Venn diagram were drawn by using the ggplot2 packages in R. The heat map was generated by using Heatmapper (http://www.heatmapper.ca/) [23].

### 2.3. GO and KEGG Pathway Enrichment Analysis of DEGs

GO analysis, which includes biological process (BP), cellular component (CC), and molecular function (MF), was conducted for features corresponding to DEGs in HBV-associated HCC samples by using the clusterProfiler [24] R package. We also used the clusterProfiler [24] R package to perform the functional enrichment analysis of DEGs in KEGG pathways. The *P*.adj < 0.05 and *q* value < 0.2 were set as the threshold for significantly enriched DEGs.

### 2.4. Construction of the Predicted PPI Network

STRING, which is a large online database of known and predicted PPI, includes direct (physical) and indirect (functional) associations [25]. First, to analyse PPI among the DEGs by using the STRING database (version 11.0), a combined score greater than 0.9 was considered significant. Second, PPI network visualization was constructed by Cytoscape [26] (version 3.8.2). Finally, to identify hub genes among DEGs, CytoHubba [27], a plug-in of Cytoscape, was used to filter out genes of the PPI network using the Maximal Clique Centrality (MCC) method.

### 2.5. Validation of Hub Gene Expression

To validate the potential role of the hub genes, we analysed the TCGA dataset which provided the RNA-Seq (level 3, HTSeq-FPKM) data along with all clinically relevant information of 424 samples [28]. The relationship between the expression level of hub genes and the clinical stages was investigated. Cox analysis was conducted to determine the relationships of hub gene expression with T classification. T classification in HCC patients was evaluated according to the tumour node metastasis (TNM) staging system [29]. The expression of hub genes in liver tumour samples and adjacent normal samples was compared using the Wilcoxon rank-sum test. Patients with liver tumours were classified into the high or low expression group based on the median value of the hub gene expression. The results are shown with violin plots and boxplots generated using the ggplot2 package in R.

### 2.6. Survival Analysis to Screen the Hub Genes

Briefly, survival analysis was performed by using the R package survival (https://cran.r-project.org/web/packages/survival/index.html) and survminer (https://cran.r-project.org/web/packages/survminer/index.html) to plot Kaplan–Meier (KM) survival curves. The Kaplan–Meier survival curves were used to represent the overall survival (OS) distributions between HCC patients with high and low expression of various hub genes. The association of gene expression with patient survival outcome was calculated using the OS time obtained from TCGA. Subsequently, receiver operating characteristic (ROC) curves were performed to further assess the results of the KM survival analysis by the R package pROC [30].

### 2.7. Immunohistochemistry-Based Validation of Hub Genes in THPA

THPA is a public database that includes over five million immunohistochemically stained tissues and cells, and it was a program supported by a grant from the Kingdom of Sweden. THPA can examine normal and carcinomic tissues by antibody proteomics and was often used to validate the expression of hub genes. Thus, this pathology tool was used to evaluate expression levels of hub genes between normal liver tissues and HCC tissues from THPA.

## 3. Results

### 3.1. Identification of DEGs in HCCs

There were 49 HCC samples and 91 normal tissues in the GSE55092 dataset. There were 70 HCC samples and 37 normal tissues in the GSE121248 dataset. By identifying the microarray results of the GSE55092 and GSE121248 datasets, 1019 upregulated and 1511 downregulated genes were identified in GSE55092, and 901 upregulated and 423 downregulated genes were identified in GSE121248. The volcano plots of each dataset are depicted for the visualization of DEGs in Figures 1(a) and 1(b). The Venn diagram shows a total of 694 overlapping DEGs in Figure 1(c). The heat map in Figure 1(d) was generated by using Heatmapper. It was drawn to show the differentially expressed genes. In this heat map, blue indicates downregulation, while red indicates upregulation.

### 3.2. KEGG and GO Enrichment Analysis of DEGs

By GO enrichment analysis, 694 overlapping DEGs were enriched for 722 biological process (BP) terms, 34 cellular component (CC) terms, and 76 molecular functional (MF) terms. Under BP terms (Figure 2(a)), DEGs were mainly enriched in the following processes: organic acid catabolic process, carboxylic acid catabolic process, and carboxylic acid biosynthetic process. For CC terms (Figure 2(b)), DEGs were primarily enriched in collagen-containing extracellular matrix, blood microparticle, and condensed chromosome kinetochore. Enrichment analysis of MF terms (Figure 2(c)) revealed that most DEGs were enriched in arachidonic acid epoxygenase activity, arachidonic acid monooxygenase activity, and monooxygenase activity. The enrichment analysis of KEGG pathways (Figure 2(d)) included 26 KEGG pathways, and most of the DEGs were significantly enriched in chemical carcinogenesis, retinol metabolism, and the p53 signalling pathway.

### 3.3. PPI Network Construction and Analysis of Hub Genes

There were a total of 694 DEGs in the PPI network, which originated from the STRING database. The PPI network was constructed to predict the interactions of common DEGs, consisting of 324 nodes and 1189 edges (Figure 3(a)). The cytoHubba plugin selected the top 10 genes (Figure 3(b)) ranked by the MCC method as hub genes, including cyclin-dependent kinase 1 (CDK1), cyclin B2 (CCNB2), cell division cycle 20 (CDC20), BUB1 mitotic checkpoint serine/threonine kinase (BUB1), BUB1 mitotic checkpoint serine/threonine kinase B (BUB1B), cyclin B1 (CCNB1), the NDC80 kinetochore complex component (NDC80), centromere protein F (CENPF), mitotic arrest deficient 2 like 1 (MAD2L1), and the NUF2 component of the NDC80 kinetochore complex (NUF2).

### 3.4. Hub Gene Expression and the Clinicopathologic Parameters of HCC Patients

The expression of 10 hub genes was analysed for its relevance to the clinicopathologic parameters of HCC patients. The expression of these genes was associated with T classification (*P* < 0.05) (Figure 4). Gene expression was increased in HCC tissues (*P* < 0.05) (Figure 5).

### 3.5. Survival Analysis of Selected Hub Genes

To further validate the prognostic value of hub genes, R was used to conduct survival analysis of the 10 genes in the 424 samples derived from the TCGA project by using the KM plotter (Figure 6). According to our KM survival curve analysis, we found that high expression of CDK1, CDC20, BUB1, BUB1B, CCNB1, NDC80, CENPF, MAD2L1, and NUF2 predicted worse survival outcome in patients with HCC (*P* < 0.05), but CCNB2 did not. Subsequently, ROC curves were generated and analysed to gain a complete view of the predictive value of the hub genes. The results showed that all hub genes were able to distinguish HCC tissues from normal liver tissue (Figure 7). Moreover, representative images indicated that the expression of hub genes was upregulated in HCC tissues (Figure 8).

## 4. Discussion

In recent years, despite great progress in the clinical therapy and pathogenesis prognosis for HCC, mortality remains unacceptably high [31]. Chronic HBV infection is the predominant aetiology of HCC, particularly in China [32]. Through performing bioinformatics analysis, we aimed to provide new insights into the molecular mechanism underlying HBV-HCC development and progression.

To overcome the disadvantages of the small sample size and heterogeneity of the studied group, we analysed several public databases, such as GEO and TCGA, through data mining approaches. In the present study, we analysed two GEO datasets (GSE55092 and GSE121248) by an integrated bioinformatics analysis. In the GSE55092 dataset, we examined 49 HCC samples and 91 normal tissues. There were 1019 upregulated and 1511 downregulated genes. In the GSE121248 dataset, we analysed 70 HCC samples and 37 normal tissues. An average of 901 upregulated and 423 downregulated genes were identified from GSE121248. We identified 694 DEGs by comparing HCC tissues and normal tissues. Next, the 694 DEGs were subjected to GO and KEGG pathway enrichment analyses. BP analysis of DEGs showed that the genes were related to the organic acid catabolic process, carboxylic acid catabolic process, and carboxylic acid biosynthetic process. The BP GO terms showed that genes were related to the organic acid catabolic process, carboxylic acid catabolic process, and carboxylic acid biosynthetic process. The CC GO terms showed that the genes were associated with the collagen-containing extracellular matrix, blood microparticle, and condensed chromosome kinetochore. The MF GO terms showed that the genes were related to arachidonic acid epoxygenase activity, arachidonic acid monooxygenase activity, and monooxygenase activity. By analysing KEGG enrichment analysis, DEGs were involved in chemical carcinogenesis, retinol metabolism, and the p53 signalling pathway. By using the STRING database, we built PPI networks and found that CDK1, CCNB2, CDC20, BUB1, BUB1B, CCNB1, NDC80, CENPF, MAD2L1, and NUF2 were hub genes.

According to the TCGA database, the expression of the 10 hub genes was found to be related to the HCC stage and was significantly higher in the tumour tissues. Further survival analyses, ROC curve analysis and representative image analysis, selected 5 hub genes, including CDK1, CDC20, CCNB1, CENPF, and MAD2L1, that were associated with early diagnosis, tumour stage, and poor outcomes of HCC.

CDK1 is a member of the serine-threonine protein kinases. Because it is crucial for mitosis, the aberrant expression of the CDK1 gene correlates with various tumours [33–35]. The study of Tian et al. [36] confirmed that miR-31/CDK1 can regulate the growth, migration, and invasion of bladder cancer. The research by Yang et al. [37] confirms that CDK1 is associated with cancer growth and the survival rate of epithelial ovarian cancer. Recent findings [38] show that CDK1 affects 5-Fu resistance in colorectal cancer. Moreover, another study reported that the CDK1/CCNB1 axis can regulate hepatocarcinogenesis [39].

A study by Cai et al. [40] suggests that CDK1 is a prognostic and therapeutic target for HBV-HCC. In our research, we performed GO function and KEGG analysis, survival analysis, ROC curve analysis, and representative image analysis of CDK1. The results from these analyses support the above conclusion. CDK1 may play a role in early diagnosis, tumour stage, and poor outcomes of HBV-HCC.

CDC20 acts as a regulating protein in the cell cycle [41]. Many studies suggest that CDC20 is overexpressed in many cancers [42]. It is related to the prognosis and progression in prostate, glioma, breast, and other cancers [43–46]. In particular, CDC20 expression is associated with the development and progression of HBV-HCC [47, 48]. By using GO function and KEGG analyses, survival analysis, ROC curve analysis, and representative image analysis of CDC20, our findings demonstrate that CDC20 may play a role in early diagnosis, tumour stage, and poor outcomes of HBV-HCC.

CCNB1, which encodes a regulatory protein involved in mitosis called CCNB1, is an influential member of the conserved cyclin B family [49]. Abnormal expression of the CCNB1 gene can influence the cell cycle and cell proliferation, leading to various malignant tumours [50–53]. The study by Zhang et al. [54] found that silencing CCNB1 can influence cell cycle, senescence, and apoptosis in pancreatic cancer. Research by Lin et al. [55] showed that overexpression of CCNB1 can enhance chondrosarcoma progression. Particularly for HCC, the growth, proliferation, migration, and invasion were strongly associated with CCNB1 [56, 57]. The study by Weng et al. [58] demonstrated that CCNB1 also has the potential to become a candidate biomarker and therapeutic target for HBV-HCC. In this study, GO function and KEGG analyses, survival analysis, ROC curve analysis, and representative image analysis of CCNB1 were performed. These findings support the above conclusion. CCNB1 plays a significant role in the early diagnosis, tumour stage, and poor outcomes of HBV-HCC.

CENPF encodes a protein that associates with the centromere-kinetochore complex and influences cell cycle, division, and differentiation [59]. It has been reported that CENPF is related to multiple kinds of malignancies such as prostate and breast cancer [60, 61]. In particular, the research of Yang et al. found that CENPF could promote the tumour growth of HCC [31]. Thus, CENPF could serve as a novel target for early diagnosis, tumour stage, and poor outcomes in HBV-HCC.

MAD2L1 is a component of the mitotic spindle assembly checkpoint [62] and has been reported to be linked to various types of cancers, such as rhabdomyosarcoma and gastric cancer [63, 64]. In parallel, MAD2L1 correlates with proliferation, progression, and metastatic risk in HBV-HCC [65, 66]. Consequently, MAD2L1 is also an important indicator of the early diagnosis, tumour stage, and poor outcomes of HCC.

In the current study, DEGs were screened between two datasets, and the TCGA database was used for the survival analysis of the hub genes. This approach decreased random errors caused by using a single dataset and improved the reliability and quality of bioinformatic analysis. However, there were also certain limitations to this study. First, a limitation of this study is the small sample size, which limits the generalization of the results. Second, because of the limitations of medical conditions in Chongming District, the 5 hub genes indicated here have not been confirmed in clinical studies. In future studies, we will collect samples in Shanghai to test hub genes by performing experiments in a clinical sample size. After clinical experiments, the associations and mechanisms of action of the candidate genes will also require confirmation by in vitro and in vivo trials.

## 5. Conclusion

In conclusion, our study identified 694 DEGs in HBV-HCC by bioinformatics analysis. DEGs provided an insight into the mechanisms of HBV-HCC and increase our understanding of the mechanisms of pathogenesis and prognosis. Based on downstream analysis, 5 hub genes, including CDK1, CDC20, CCNB1, CENPF, and MAD2L1, that could play a critical role in the early diagnosis, tumour stage, and poor outcomes of HBV-HCC were identified.

## Figures and Tables

**Figure 1:** Identification of DEGs in HBV-associated HCC. (a, b) Two volcano plots showing all the expressed genes from GSE55092 and GSE121248. (c) Venn diagram for the overlapping DEGs by R. (d) Heat map of 694 overlapping DEGs. Blue represents downregulated genes, and red represents upregulated genes. Each column represents one dataset, and each row represents one gene. DEGs: differentially expressed gene.

**Figure 2:** KEGG and GO enrichment analysis of DEGs. (a–d) DEGs: differentially expressed genes; GO: Gene Ontology; BP: biological process; CC: cellular component; MF: molecular function; KEGG: Kyoto Encyclopedia of Genes and Genomes.

**Figure 3:** PPI network construction and analysis of hub genes. (a) The most significant module was obtained from the PPI network with 324 nodes and 1189 edges. (b) The hub genes were selected from the PPI network using the cytoHubba plugin. DEGs: differentially expressed genes; PPI: protein–protein interaction.

**Figure 4:** Clinicopathologic parameters of HCC patients associated with T classification: (a) CDK1 (*P* = 0.001); (b) CCNB2 (*P* = 0.011); (c) CDC20 (*P* = 0.019); (d) BUB1 (*P* = 0.003); (e) BUB1B (*P* = 0.004); (f) CCNB1 (*P* = 0.007); (g) NDC80 (*P* = 0.005); (h) CENPF (*P* = 0.003); (i) MAD2L1 (*P* = 0.001); (j) NUF2 (*P* = 0.004). CDK1: cyclin-dependent kinase 1; CCNB2: cyclin B2; CDC20: cell division cycle 20; BUB1: BUB1 mitotic checkpoint serine/threonine kinase; BUB1B: BUB1 mitotic checkpoint serine/threonine kinase B; CCNB1: cyclin B1; NDC80: NDC80 kinetochore complex component; CENPF: centromere protein F; MAD2L1: mitotic arrest deficient 2 like 1; NUF2: NUF2 component of NDC80 kinetochore complex.

**Figure 5:** Expression of various genes in the tumour samples and normal samples. “Tumour free” represents the normal tissue, and “With tumour” represents the tumour samples: (a) CDK1 (*P* = 0.004); (b) CCNB2 (*P* = 0.003); (c) CDC20 (*P* = 0.002); (d) BUB1 (*P* = 0.004); (e) BUB1B (*P* = 0.003); (f) CCNB1 (*P* = 0.004); (g) NDC80 (*P* = 0.017); (h) CENPF (*P* = 0.004); (i) MAD2L1 (*P* < 0.001); (j) NUF2 (*P* = 0.009). CDK1: cyclin-dependent kinase 1; CCNB2: cyclin B2; CDC20: cell division cycle 20; BUB1: BUB1 mitotic checkpoint serine/threonine kinase; BUB1B: BUB1 mitotic checkpoint serine/threonine kinase B; CCNB1: cyclin B1; NDC80: NDC80 kinetochore complex component; CENPF: centromere protein F; MAD2L1: mitotic arrest deficient 2 like 1; NUF2: NUF2 component of NDC80 kinetochore complex.

**Figure 6:** Overall survival (OS) curves of the 10 hub genes. Overall survival (OS) curves by high and low expression of various genes in HCC patients: (a) CDK1; (b) CCNB2; (c) CDC20; (d) BUB1; (e) BUB1B; (f) CCNB1; (g) NDC80; (h) CENPF; (i) MAD2L1; (j) NUF2. CDK1: cyclin-dependent kinase 1; CCNB2: cyclin B2; CDC20: cell division cycle 20; BUB1: BUB1 mitotic checkpoint serine/threonine kinase; BUB1B: BUB1 mitotic checkpoint serine/threonine kinase B; CCNB1: cyclin B1; NDC80: NDC80 kinetochore complex component; CENPF: centromere protein F; MAD2L1: mitotic arrest deficient 2 like 1; NUF2: NUF2 component of NDC80 kinetochore complex.

**Figure 7:** Receiver operating characteristic curves for the 10 hub genes: (a) CDK1 (AUC = 0.977, CI = 0.962–0.992); (b) CCNB2 (AUC = 0.976, CI = 0.962–0.989); (c) CDC20 (AUC = 0.980, CI = 0.967–0.993); (d) BUB1 (AUC = 0.969, CI = 0.953–0.985); (e) BUB1B (AUC = 0.961, CI = 0.942–0.981); (f) CCNB1 (AUC = 0.981, CI = 0.969–0.993); (g) NDC80 (AUC = 0.982, CI = 0.967–0.996); (h) CENPF (AUC = 0.979, CI = 0.967–0.991); (i) MAD2L1 (AUC = 0.953, CI = 0.93–0.976); (j) NUF2 (AUC = 0.983, CI = 0.972–0.993). CDK1: cyclin-dependent kinase 1; CCNB2: cyclin B2; CDC20: cell division cycle 20; BUB1: BUB1 mitotic checkpoint serine/threonine kinase; BUB1B: BUB1 mitotic checkpoint serine/threonine kinase B; CCNB1: cyclin B1; NDC80: NDC80 kinetochore complex component; CENPF: centromere protein F; MAD2L1: mitotic arrest deficient 2 like 1; NUF2: NUF2 component of NDC80 kinetochore complex.

**Figure 8:** Representative histological images from the Human Protein Atlas database (THPA, https://www.proteinatlas.org/). Normal liver tissue with staining for CDK1 was obtained from a female subject aged 32 years (patient ID: 1846; staining: not detected; intensity: negative; quantity: none; location: none; magnification: not available), and HCC tissue was obtained from a female patient aged 73 years (patient ID: 2279; staining: medium; intensity: strong; quantity: <25%; location: cytoplasmic/membranous nuclear; magnification: not available). Normal liver tissue with staining for CCNB2 was obtained from a male subject aged 55 years (patient ID: 2429; staining: not detected; intensity: negative; quantity: none; location: none; magnification: not available), and HCC tissue was obtained from a female patient aged 52 years (patient ID: 2399; staining: medium; intensity: moderate; quantity: 75%-25%; location: cytoplasmic/membranous; magnification: not available). Normal liver tissue with staining for CDC20 was obtained from a male subject aged 67 years (patient ID: 1720; staining: not detected; intensity: negative; quantity: none; location: none; magnification: not available), and HCC tissue was obtained from a male patient aged 57 years (patient ID: 1175; staining: medium; intensity: strong; quantity: <25%; location: cytoplasmic/membrane nuclear; magnification: not available). Normal liver tissue with staining for CCNB1 was obtained from a female subject aged 32 years (patient ID: 1846; staining: not detected; intensity: negative; quantity: none; location: none; magnification: not available), and HCC tissue was obtained from a female patient aged 65 years (patient ID: 937; staining: medium; intensity: strong; quantity: <25%; location: cytoplasmic/membranous; magnification: not available). Normal liver tissue with staining for CENPF was obtained from a female subject aged 32 years (patient ID: 1846; staining: not detected; intensity: negative; quantity: none; location: none; magnification: not available), and HCC tissue was obtained from a female patient aged 65 years (patient ID: 937; staining: medium; intensity: strong; quantity: <25%; location: cytoplasmic/membranous; magnification: not available). Normal liver tissue with staining for MAD2L1 was obtained from a male subject aged 55 years (patient ID: 2429; staining: not detected; intensity: negative; quantity: none; location: none; magnification: not available), and HCC tissue was obtained from a female patient aged 67 years (patient ID: 3334; staining: medium; intensity: moderate; quantity: >75%; location: cytoplasmic/membranous; magnification: not available). CDK1: cyclin-dependent kinase 1; CCNB2: cyclin B2; CDC20: cell division cycle 20; CCNB1: cyclin B1; NDC80: NDC80 kinetochore complex component; CENPF: centromere protein F; MAD2L1: mitotic arrest deficient 2 like 1; NUF2: NUF2 component of NDC80 kinetochore complex.

## Data Availability

The gene expression profiling data supporting this study are from previously reported studies and datasets, which have been cited. The processed data are available at the Gene Expression Omnibus (GEO) database.
